This article has been retracted.

# Can Information Intervention Enhance Consumers' Purchase Intentions of Organic Agricultural Products? A Choice Experiment Based on Organic Milk

**DOI:** 10.1155/2022/1256796

**Published:** 2022-03-31

**Authors:** Chang Dou, Lihang Cui, Cuixia Li

**Affiliations:** School of Economics and Management, Northeast Agricultural University, Harbin, Heilongjiang 150030, China

## Abstract

Despite the current rapid growth of organic agriculture, the problem of low demand for organic agricultural products persists in China, and the consumption space warrants improvement. Exploring consumers' preferences for organic agricultural products and increasing their purchase intentions are of utmost significance to promote organic agricultural production. Thus, this study takes organic milk, which accounts for 58% of China's organic processed agricultural products in sales, as the research object, and uses a choice experiment to investigate the influence of consumers on the purchase intention of organic milk under the intervention of environmental protection information and quality and safety information. The main research results revealed that both environmental protection information and quality and safety information have significantly increased consumers' willingness to purchase and that quality and safety information has increased more than environmental protection information.

## 1. Introduction

To fulfill people's rising consumer demand, improve the quality of agricultural products, and protect the agricultural production environment, the Chinese government is actively promoting and developing organic agriculture throughout the country. Per the latest data from China's Organic Product Certification and Organic Industry Development (2020), the output value of China's organic agricultural products increased from 129.9 billion yuan to 167.2 billion yuan during 2015–2019, with an average annual growth rate of 12.55%. Despite the abovementioned accomplishments, China's organic agricultural products are still facing the problems of inadequate demand and low consumer purchasing intention. With improved living standards and health concepts, consumers are paying ever more attention to organic agricultural products, and the development of the organic agricultural product market has gradually transitioned from being driven by production to being driven by demand [1]. In 2018, China's organic agricultural product sales amounted to 8.1 billion euros, accounting for 8% of the global total and making China the world's third-largest consumer of organic food. Although, in absolute terms, China has become the third-largest single market for organic agricultural products, regarding relative volume, the consumption space of organic agricultural products in China still needs to be tapped, and consumers' purchase intentions still need to be improved. This is primarily reflected in three aspects. First, the percentage of organic agricultural products is low in China. The consumption of organic agricultural products in China only accounts for 3.65% of the total consumption of agricultural products, which is much smaller than developed countries such as the United States (6%), Denmark (11.5%), Switzerland (9.9%), and Sweden (9.6%). Second, the per-capita consumption of organic agricultural products in China is not high. Besides, per-capita sales of organic agricultural products in China is 48.77 yuan, which is less than the global average of 100 yuan. Third, the inadequate scale on the production side is due to deficient consumption on the consumer side. Currently, the output value of organic agricultural products only accounts for 1.5% of the total agricultural output value. Meanwhile, China's organic farming area only accounts for 0.85% of agricultural lands, far below the global average of 1.5%.

Primarily, consumers buy organic agricultural products for food safety, health, and the environment. Han [1] claimed that Chinese urban residents make purchase decisions based on price information, nutrition, and safety of organic agricultural products. Nevertheless, most individual demands are dormant for most of the time, and the general lack of cognition of organic agricultural products by most consumers in China limits the stimulation of demand. Cognition is the process of recognizing objective things and acquiring knowledge. The research on consumer behavior demonstrated that consumers form knowledge and understanding and evaluate products through cognitive activities, which, in turn, generate preferences and eventually transform them into buying behavior [2]. Cognition affects consumers' willingness to pay for organic agricultural products [3, 4].

Although the consumption of organic agricultural products has snowballed in developing countries, their consumers' cognition of organic agricultural products is limited [5]. Wang et al. [6] surveyed Shayibake district, Urumqi city, and reported that consumers have unsatisfactory awareness of organic vegetables and 74% of consumers do not understand the concept of organic vegetables very well or at all; besides, the current consumers' cognition of organic vegetables is not high. Ma and Qin [7] examined Beijing's urban residents and reported that residents have inadequate cognition of organic agricultural products. Then, information intervention has become one of the crucial ways to enhance consumers' purchase intentions of organic agricultural products through the cognitive process. Magistris and Gracia [8] established that information intervention would enable consumers to have a better understanding of organic food and increase their cognitive level, thereby promoting consumer purchases. Yin et al. [9] reported that under information intervention, consumer cognition was enhanced, which markedly increased the willingness to pay for organic tomatoes [9]. To date, limited studies have examined the issue of information intervention to increase purchase intention, and there is no difference in research on the impact of different information interventions on purchase intention. Thus, this study aims to use information intervention as a breakthrough point to perform information intervention on the purchase intention of organic agricultural products and solve the problem of consumer purchasing intention of organic agricultural products, which is of utmost significance for expanding organic agricultural production.

## 2. Theoretical Framework

Consumers purchase organic agricultural products based on their needs for food safety, health, and environmental protection; however, most individual needs are dormant for most of the time. At a specific time, certain cognitions are activated through sensory input, which can induce needs and trigger cognitive awareness [10]. The general lack of awareness of most Chinese consumers of organic agricultural products limits the demand stimulation. The creation of sensory stimulation through information intervention can activate specific cognition, induce demand, and finally influence consumer behavior.

Per the three-dimensional arousal theory, arousal can be summarized into three processes: (i) the general internal stimulus arousal due to physiological conditions, (ii) the “emotional arousal” system (the demand is triggered by the emotional process, which leads to defense reactions and negative emotions), and (iii) the arousal of needs in the cognitive process, which is the most important one in mature individuals. Consumers' processing of information is affected by their characteristics and the external environment, and various pieces of information from the outside world create their basic cognition of the problem through the processing of the consumer's brain [11]. Through cognitive awakening, the awareness of needs is triggered, potential needs into attitudes and beliefs is transformed, and behavioral tendencies are formed[10, 12].

Although the purchase intention of organic agricultural products is also influenced by factors such as price, income, trust, and information asymmetry [7, 13, 14], how to overcome the lack of cognitive awareness of potential consumer demand is an urgent issue in the current consumption of organic agricultural products. Based on the abovementioned literature and theoretical explanations, through cognitive awakening, constructing the transmission mechanism of information is critical to improve the purchase intention of organic agricultural products, where high-quality safety level and environmental protection are the leading characteristics of organic agricultural products [14–16]. Agricultural products have the attribute of “trustworthy goods” [17], and it is challenging to judge their quality. With information asymmetry and deficient government supervision, consumers can only make purchase decisions through subjective judgments. Nevertheless, organic agricultural products can pass information to consumers through organic certification and quality traceability systems to eliminate information asymmetry and ensure food quality and safety [18]. Moreover, organic agricultural products have the attributes of public goods. The consumption behavior leads to ecological environment optimization, and consumers can reap the benefits of environmental protection without paying the price [19]. However, consumers have inadequate access to food safety information or knowledge [20], and it is hard to acquire comprehensive environmental knowledge, which results in a low level of environmental cognition [21]. The quality and safety information and environmental protection information are input into the human brain, and through the cognitive awakening process, it triggers cognitive awareness and stimulates consumers' needs for food safety, health needs, and environmental protection, activating these latent demands in a dormant state and finally affecting purchase intention (Figure 1).

This study uses environmental protection information and quality and safety information as different pieces of intervention information to determine whether the purchase intention of organic agricultural products is improved under the information intervention and whether differences exist in the influence of different information interventions on the purchase intention of organic agricultural products. In addition, this study attempts to use organic milk as the research object for the following reasons: (i) organic milk is a crucial organic agricultural product, with its sales accounting for 58% of organic processed products; (ii) as the national income level increases, residents' health awareness is increasing gradually, and the awareness of obtaining protein from milk to enhance resistance has increased; in addition, organic milk, as a representative of high-quality milk, can better cater to consumption trends.

Hence, this study adopts the method of choice experiments and analyzes the influence of consumers on the purchase intention of organic milk under different pieces of intervention information through the random parameter logit (RPL) model. Of note, this is of great practical significance for expanding consumer demand for organic agricultural products, promoting the development of organic agriculture in China and increasing domestic demand.

## 3. Experimental Design

### 3.1. Information Intervention and Experimental Projects

To examine the impact of environmental protection information and quality and safety information on the purchase intention of organic milk, we designed three project experiments. Random sampling surveys were conducted in shopping malls, supermarkets, and other places in Harbin, and each subject was tested individually. In the first project experiment, participants were divided into three groups—*a*, *b*, and *c*—which were different groups. Participants in group *a* did not accept any information intervention and conducted choice experiments; participants in group *b* conducted choice experiments after receiving environmental protection information; participants in group *c* conducted choice experiments after receiving quality and safety information. While group *a* was the control group, groups *b* and *c* were the experimental groups. The experiment implementer delivered the following environmental protection information to participants through oral notification: the soil, air, and water sources in the organic dairy farm must fulfill the organic agricultural production standards of the relevant country or region, including heavy metals in the soil and carbon emissions in the air. Of note, strict implementation standards have been set for quantity and water quality. Besides, we conveyed the following quality and safety information through oral notification: ① in the process of organic production and processing, use of synthetic chemical substances such as chemical fertilizers, pesticides, hormones, growth regulators, feed additives, and food additives is sternly prohibited, and packaging, storage, and transportation must strictly comply with the relevant standards of organic food; ② organic milk is produced in compliance with national or regional organic product production standards, abides by the organic food quality and safety production system, and is certified by a third-party organic certification body.

As the three groups of participants *a*, *b*, and *c* in the first project experiment comprised completely different people, even if participants' demographic characteristics and other factors that influence purchase intentions are controlled, the experimental results could still be biased. Thus, after the first project experiment, we continued to implement the second and third project experiments. In the second project experiment, participants were randomly selected; in this experiment, participants first conducted the choice experiment without any information intervention, which was group *d*. Subsequently, the choice experiment was conducted again after the environmental protection information intervention, which was group *e*.

The third project experiment was similar to the second, and random sampling of participants was performed. First, a choice experiment was conducted when participants did not perform information intervention, which was group *f*. Then, after intervening in quality and safety information, a choice experiment was implemented, which was group g.

Besides the choice experiment, before the experiment, participants' demographic characteristics (including gender, age, education level, and monthly income), family characteristics (whether there were any elders aged >60 years in the family and whether there were children aged >1 year in the family), “trust in organic milk,” and “the experience of paying attention to organic milk” were also investigated.

This experiment was conducted by members of the animal husbandry economic management team of the School of Economics and Management of Northeast Agricultural University. Each experiment required that the experiment ended when the number of experimenters reached 100. Thus, the number of subjects in each group of each experiment was 100. The experiment locations were shopping malls and supermarkets in Harbin. The experiment duration was June 10–24, 2021, as shown in Table 1.

### 3.2. Choice Experimental Attributes and Levels

Too many attributes will increase the information load of the experiment, which would lead to bias due to consumer fatigue or limited cognitive ability; conversely, too few attributes would lead to simulation distortion or missing variables [22]. Based on the existing literature and the demand for organic milk in the current market, we set the organic certification mark, brand location, raw milk origin, and price as the attributes of organic milk (Table 2). The attributes and levels of organic milk were specifically set as follows:

#### 3.2.1. Organic Certification Mark

Organic milk is a milk product produced per organic production standards and specifications and has passed the organic certification of a third-party certification body. The organic certification mark on the organic milk packaging is the most crucial feature differentiating organic milk from ordinary milk. The pertinent literature uses the organic certification mark as one of the attribute characteristics of organic agricultural products. In this study, we set the attributes of the organic certification mark into two levels because organic milk products on the market have either passed Chinese organic certification or the organic certification of other countries or regions. Thus, we set the level as Chinese organic certification mark and foreign organic certification mark.

#### 3.2.2. Brand Location

Influenced by the melamine incident, consumers' trust in domestic dairy products has been undermined, making consumers prefer foreign dairy products. The existing studies have demonstrated that consumers prefer foreign brands of organic milk to domestic brands. Of note, consumers pay particular attention to the brand attributes of organic milk [23]. Hence, we set the brand location attribute as two levels—Chinese (domestic) brands and foreign brands.

#### 3.2.3. Origin of Raw Milk

Consumers may prefer local or domestic agricultural products, as well as prefer agricultural products from foreign origins [24–26]. The origin plays a vital role in the selection of agricultural products. This study divides the origin of raw milk into two levels: China (domestic) and foreign.

#### 3.2.4. Price

In the choice experiment design, the price is usually set to five levels [27]. Based on the actual market research, we set the price of ordinary milk (or nonorganic milk) that does not contain organic attributes at 3.80 yuan/250 mL. The floating price was set according to the aforementioned price [28]. Based on the previous research [29] on the choice experimental price setting of organic milk, we set a 40% price fluctuation.

### 3.3. Orthogonal Experimental Design

Per the attributes and levels designed in Table 2, a full factorial design can form 2 × 2 × 2 × 5 = 100 organic milk options. If these options are combined in pairs to form a selection set, there will be 780 selection sets. So many choices will cause a great cognitive burden on participants, resulting in a lower response rate and lower experimental reliability [30]. Thus, it is essential to use an orthogonal experimental design to decrease the number of choices faced by participants. The orthogonal test contains all levels of all factors. All combinations of levels in any two columns appear so that all levels of information of any two factors and all levels of combination information are not omitted. Therefore, the orthogonal experimental design can represent a comprehensive experimental design. In this study, we used SAS ONDEMAND FOR ACADEMICS online statistical analysis software to perform experimental design and determined 18 selection sets. Each selection set contained choices *A*, *B*, and a no-choice *C*, which are combined by different attributes. Meanwhile, according to the program design, 18 selection sets were divided into three groups, and each group contained six selection sets. This way, each participant could randomly select one group and conduct six selection experiments in the selected combination, which markedly reduced the experimental pressure of participants to ensure the validity of the experiment.  Table 3 shows an example of the selection set.

## 4. Model Construction and Variable Settings

### 4.1. Model Construction

Lancastrian demand theory stipulates that consumers pay attention to and consume the product's objective characteristics rather than the product itself when selecting a product bundle. That is to say, consumers cannot obtain utility from the commodity itself but from the attribute characteristics of the commodity (Lancaster et al., 1966) [31].

The demand for a certain commodity is the activity of separating the characteristic attributes from the commodity. In this study, organic milk is described as a commodity with organic certification marks, brand locations, origin of raw milk, and price characteristics. Assuming that a consumer *n* obtains the commodity utility from consumption option *j* in the consumption decision of organic milk in the selection scenario *s*, the consumer's utility function for organic milk can be expressed as follows:

(1) $$\begin{array}{c} U_{nsj}=V_{nsj}+\varepsilon_{nsj}. \end{array}$$

Typically, *U*_*snj*_ is divided into two parts: the observable component *V*_*nsj*_ of the utility and the unobservable component *ε*_*nsj*_ of the utility.

The observable component *V*_*nsj*_ of the utility can be depicted by a linear combination of the attribute characteristics of the option and the estimated value of the parameter:

(2) $$\begin{array}{c} V_{nsj}=\sum_{k=1}^{K}\beta_{k}x_{nsjk}. \end{array}$$

Here, *x*_*nsjk*_ denotes the vector of *k* attributes of option *j*, and *β*_*k*_ denotes the parameter to be estimated.

Consumer *n* chooses option *j* in the selection scenario *s* based on *U*_*nsj*_ > *U*_*nsq*_ (for any *j* ≠ *q*); the probability of consumer *n* choosing option *j* in the selection scenario *s* can be expressed as follows:

(3) $$\begin{array}{c} P_{nsj}=\text{prob}\left(U_{nsj}>U_{nsq};\forall q\in J_{ns},q\neq j\right)\\ =\text{prob}\left(V_{nsj}+\varepsilon_{nsj}>V_{nsq}+\varepsilon_{nsq};\forall q\in J_{ns},q\neq j\right)\\ =\text{prob}\left(\varepsilon_{nsq}-\varepsilon_{nsj}<V_{nsj}-V_{nsq};\forall q\in J_{ns},q\neq j\right). \end{array}$$

Here, *J*_*ns*_ implies that consumer *n* has *J* selectable options in the selection scenario *s*, that is, the number of options in each selection scenario is *J*.

If it is assumed that the residual items satisfy both the independent and identical distribution condition and the extreme value distribution of type I, then the first-order difference of the residual items satisfies the logical distribution. At this time, the conditional logit model of consumer *n* selected option *j* determined by (1) and (4) can be expressed as follows:

(4) $$\begin{array}{c} P_{nsl}=\frac{\exp\left(\beta_{n}Z_{nsj}\right)}{\sum_{j}\exp\left(\beta_{n}Z_{nsj}\right)},\;\left(j\in J_{ns}\right). \end{array}$$

Each consumer has his/her own parameter *β*_*n*_ information and unobserved effect *ε*_*nsj*_ information; however, the consumer information cannot be directly observed. Nonetheless, it can be expressed by the probability density function *f(β*_*n*_). Thus, the unconditional selection probability given by observing *Z*_*nsj*_ is as follows:

(5) $$\begin{array}{c} P_{nsj}=\int \frac{\exp\left(\beta_{n}Z_{nsj}\right)}{\sum_{j}\exp\left(\beta_{n}Z_{nsj}\right)}f\left(\beta_{\text{n}}\right),\;\left(j\in J_{ns}\right). \end{array}$$

Of note, formula (5) is the RPL.

The RPL breaks through the assumptions of the homogeneity of individual preferences and the “independence of irrelevant options” (IIA), and, at the same time, relaxes the constraints on the normal distribution of random utility *ε*_*ij*_. A significant difference between the RPL model and the traditional logit model is that it can measure heterogeneous individuals [32].

### 4.2. Control Variable Selection and Assignment

The main advantages of the experimental method are reliability and controllable characteristics [33]. The experimental design allowed us to control the relevant information of participants and avoid individual differences from affecting the experiment.

The control variables in this study included the following three aspects: (i) Demographic characteristics, that is, gender, age, education level, personal monthly income, and family characteristics (whether there are elderly people aged >60 years in the family or whether there are children aged >1 year in the family); these personal characteristics and special groups of people in the family will affect buying behavior [34, 35]. (ii) Trust in organic milk. Trust exerts a crucial impact on the purchase behavior of organic agricultural products. Consumers with high trust are more likely to have high purchase behavior [36]. Based on the characteristics of organic milk “trusted goods,” the key to purchase is trust, and trust in organic milk is adequate to change consumers' purchase decisions [37, 38]. Before the experiment, the subjects were asked, “Compared to ordinary milk, do you trust organic milk more?” The answers were assigned a value of 1–5, representing “completely distrusted,” “relatively distrusted,” “general trust,” “relatively trusted” and “full trust.” (iii) The experience of paying attention to organic milk. Consumers' final decision to purchase a specific product requires continuous accumulation and full exchange of information [11]. At this stage, various social media have become the foremost media for people to transmit information, and their reports and introductions on organic milk might motivate people to further understand. Thus, consumers with a history of paying attention to organic milk might be more willing to buy than consumers who have not. Before the experiment, participants were asked, “Have you ever paid attention to organic milk?” The answers were assigned a value of 1 or 0, with 1 for “Yes,” and 0 for “No.”

In this study, the price is represented by the actual price selected by the consumer, and other variables are represented by dummy variables (Table 4)

## 5. Data Analysis and Results

### 5.1. Descriptive Statistical Analysis

Table 5 presents the basic statistical characteristics of control variables. The average gender was 0.43–0.55, suggesting that the gender distribution of each group is balanced. The age, education level, and personal monthly income of each group are consistent with the normal distribution, which guarantees the consistency of the surveyed groups among various groups. The proportion of elderly people aged >60 years in each group of households was 30%–48%. The proportion of families with children aged >1 year was 57%–72%. The average trust level of each group of participants in organic milk was >3.5 and <4, suggesting that the subject group is between “general trust” and “relatively trusted” in organic milk. The average value of the experience of paying attention to organic milk in each group was 0.18–0.26, suggesting that the proportion of people in each group who have had the experience of paying attention to was 18%–26%.

### 5.2. Empirical Analysis Results of the Impact of Different Information Interventions on Purchase Intention (the First Project Experiment)

As shown in Table 6, the estimation results revealed that the significance of the model improved after consumer intervention in environmental protection and quality and safety information, increasing the model's interpretation ability significantly. Quality and safety information exerts a more significant impact on purchase intention than environmental protection information.

When consumers receive environmental protection information, the results showed that the organic certification mark, brand location, and origin of raw milk variable coefficients increased significantly. Besides, the price was significant at the 1% significance level, and the coefficient was negative, suggesting that compared with no information intervention, environmental protection information increased the utility of consumers and increased their purchase intentions. Consumers' purchase intentions of foreign organic certification marks, foreign brands, and foreign raw milk increased markedly after the intervention of environmental protection information. Price exerted a restraining effect on purchase intention, but after the intervention of environmentally friendly information, the restraining effect of price was reduced, and the reduction in utility due to each increase in price was smaller than that of the situation without information intervention.

After being interfered with by quality and safety information, the results revealed that the organic certification mark coefficient increased by 52%, the brand location coefficient increased by 148%, and the raw milk production area coefficient increased by 38%. That is to say, the intervention of quality and safety information markedly increased the utility of consumers and made consumers more willing to buy organic milk with foreign organic certification marks, from foreign brands, and made from foreign raw milk. After the intervention of quality and safety information, the price coefficient increased; that is, the quality and safety information made consumers less sensitive to prices, and the impact of prices on consumers' purchase intentions was reduced.

Under information intervention, quality and safety information exerted a more significant impact on the improvement of consumer utility than environmental protection information. From the perspective of the organic certification mark, brand location, origin of raw milk, and price coefficients in the control and experimental groups, after receiving information intervention, the coefficient in group *c* was greater than that in group *b*, and the significance of the brand and raw milk-producing area of group *c* was greatly improved compared with that of group *b*. Thus, consumers interfered by quality and safety information were more willing to buy than consumers interfered by environmental protection information. In addition, consumers under quality and safety information were more willing to buy organic milk with foreign organic certification marks, from foreign brands, and made from foreign raw milk than under environmental protection information, and the effect of price also weakened under the quality and safety information.

Among the control variables, gender, age, and education level were significant under the information intervention, and the significance levels were 1%, 10%, and 5%, respectively. The significance level of personal monthly income after the information intervention increased significantly, showing that women and consumers with younger age, at a higher education level, and in a higher-income group were able to increase the purchase intention of organic milk more through information intervention. Moreover, the trust in organic milk affected purchase intention at the 5% significance level, and consumers who trust more in organic milk are more likely to buy organic milk. The experience of paying attention to organic milk was not significant in groups *a* and *b*, and the significance level was 10% in group *c*, suggesting that the experience of paying attention to organic milk has limited influence on purchase intention.

### 5.3. Experimental Test of the Impact of Information Intervention on Purchase Intention

In the first experiment, groups *a*–*c* had different groups of people. Although we added control variables that affect their purchase intentions owing to the influence of individual heterogeneity, errors were still unavoidable. Hence, we continued adding the second and third project experiments. In the second project experiment, groups *d* and *e* were of the same population, and groups *f* and *g* in the third project experiment were of the same population. Meanwhile, the second and third project experiments did not have the same number of participants. In addition, environmental protection information intervention was conducted on the second project experiment, and quality and safety information intervention was conducted on the third project experiment to validate whether the information intervention in the same subject group would affect purchase intention.

As shown in Table 7, in the second project experiment, after the intervention of environmental protection information, the coefficients of the four attributes of organic milk increased, suggesting that environmental protection information increased purchase willingness.

In the third project experiment, after the intervention of quality and safety information, the coefficients of the four attributes of organic milk increased, suggesting that the quality and safety information also increased the purchase intention of organic milk. Nevertheless, the increase in purchase intention obtained in the second and third project experiments after the information intervention was smaller than that in the first project experiment; this could be because the second and third project experiments were two choice experiments by the same group of participants before and after the information intervention, which caused interference and fatigue. In such a scenario, after the intervention of environmental protection information and quality and safety information, the test group still showed a stronger purchasing intention, indicating the validity of the first project experimental result.

## 6. Conclusions and Suggestions

This study took the choice experiment as the main method and used the RPL model to estimate and investigate the influence of consumers on the purchase intention of organic milk under the intervention of environmental protection and quality and safety information. The abovementioned research showed the following.

First, both the environmental protection information intervention and the quality and safety information intervention significantly improve consumers' purchase intentions, and the quality and safety information has a greater increase in the purchase intention of organic milk than the environmental protection information.

Second, irrespective of whether information intervention is performed, consumers have shown a preference for foreign organic certification marks, foreign brands, and foreign raw milk. Information intervention will further increase consumers' preference for foreign organic certification marks, foreign brands, and foreign raw milk. The organic certification mark exerts the highest impact on purchase intentions.

Third, after information intervention, the effect of price on purchase intention is reduced; that is to say, after information intervention, every increase in price by one unit decreases the degree of reduction in consumer utility, and the sensitivity of price to the impact of purchase intention decreases.

Fourth, women, younger groups, and consumers with higher education levels and higher incomes are more likely to increase their purchase intentions of organic milk through information intervention. Meanwhile, notwithstanding information intervention, trust in organic milk affects purchase intention markedly.

Based on the abovementioned research conclusions, this study proposes the following suggestions for the government to increase the purchase intention of organic milk:

First, fortify the promotion of organic milk and increase consumer awareness. ① Expand the scope of publicity and promotion. Promote organic milk knowledge through online media, TV, and other online media or through offline methods such as organic milk science lectures and community knowledge forums. ② Conduct multiangle publicity. Enhance consumers' knowledge about quality and safety and environmental protection, particularly on quality and safety, and promote consumers' awareness of organic milk.

Second, enhance consumers' market recognition of domestic organic milk. ① Improve the recognition of organic certification marks. Augment the supervision of the certification and accreditation of China's organic food production certification marks, strengthen the effective supervision of third-party certification agencies, and improve the authority and international influence of China's organic certification marks. ② Reinforce residents' trust in domestic brands and domestic milk sources. Regarding policies, we will promote the high-quality development of domestic brands, encourage dairy companies to develop organic milk source bases, promote the construction of high-quality milk source bases, and toughen the supervision of the overall organic milk industry chain.

Finally, gradually decrease the cost of organic milk production. ① Augment support for organic milk production enterprises. Regarding policies, organic production enterprises are given preferential treatment in finance, taxes, and insurance, and efforts are made to decrease the cost of production factors in organic production, such as land cost. ② Improve production efficiency. Effectively guide the enterprise's factor allocation in terms of input and output, promote the production and management mode that combines production, education and research, and promote the enhancement of production efficiency.

## Figures and Tables

**Figure 1:** The influence mechanism of information intervention on the purchase intention of organic agricultural products.

**Table 1:** Experimental items, experimental groups, and information intervention.

Experimental project	The first project experiment			The second project experiment		The third project experiment	
Experimental group	*a*	*B*	*C*	*d*	*e*	*f*	*g*
Information intervention content	No	Environmental protection information	Quality and safety information	No	Environmental protection information	No	Quality and safety information
Number of subjects	100	100	100	100	100	100	100
Remark	*a*, *b*, and c are different groups			*d* and *e* are the same group		*f* and *g* are the same group	

**Table 2:** Attributes and levels of organic milk.

Attributes	Levels	Attribute description
Organic certification mark	Chinese organic certification mark	Organic certification mark displayed on organic milk packaging
	Foreign organic certification mark	
Brand location	Chinese brand	Refers to the place where the brand of organic milk belongs to
	Foreign brand	
Origin of raw milk	China	Refers to where the raw milk of organic milk belongs to
	Foreign	
Price(yuan/250 ml)	3.80	Sales price of organic milk
	5.32	
	7.45	
	10.43	
	14.6	

**Table 3:** Examples of selection sets.

Attributes	*A*	*B*	*C*
Organic certification mark	Foreign organic certification mark	Chinese organic certification mark	No choice
Brand location	Chinese brand	Foreign brand	
Origin of raw milk	China	Foreign	
Price	14.6 yuan/250 ml	10.43yuan/250 ml	
Your choice	□	□	□

**Table 4:** Variable representation and assignment.

Variables	Variable representation	Variable assignment
Organic certification mark	Certf	Foreign organic certification mark = 1; Chinese organic certification mark = 0
Brand location	Brand	Foreign brand = 1; Chinese brand = 0
Origin of raw milk	Origin	Foreign = 1; China = 0
Price	Price	Price = 3.80￥/250 ml; 5.32￥/250 ml; 7.45￥/250 ml; 10.43￥/250 ml; 14.6￥/250 ml
Gender	Gen	female = 1; male = 0
Age	Age	(0,18] = 1; (18, 25] = 2; (25, 35] = 3; (35, 50] = 4; (50, 60] = 5; (60, +∞) = 6
Education	Edu	Elementary school and below = 1; junior high school = 2; high school or technical secondary school = 3; Junior college = 4; undergraduate = 5; masters degree and above = 6
Personal monthly income(yuan)	Income	(0, 2000] = 1; (2000, 4000] = 2; (4000, 6000] = 3; (6000, 8000] = 4; (8000, 10000] = 5; (10000, +∞] = 6
Elderly people over 60 years old in the family	n_elder	yes = 1; no = 0
Children over 1 year old in the family	n_child	yes = 1; no = 0
Trust in organic milk	Trust	“Completely distrusted” = 1, “relatively distrusted = 2”, “general trust = 3”, “relatively trusted = 4” and “full trust = 5”
The experience of paying attention to organic milk	Attention	yes = 1; no = 0

**Table 5:** Basic characteristics of samples of each project in the choice experiment.

Variables	The first project						The second project		The third project	
	Group a		Group b		Group c		Group *d* or e		Group *f* or g	
	Average	SD	Average	SD	Average	SD	Average	SD	Average	SD
Gender	0.52	0.499	0.47	0.499	0.5	0.5	0.55	0.497	0.43	0.495
Age	3.45	1.32	3.34	1.04	2.90	1.77	3.63	2.10	3.51	1.48
Education	2.61	0.96	3.02	1.09	2.58	0.99	2.88	1.35	2.90	1.02
Personal monthly income(yuan)	2.01	0.89	2.42	0.97	2.63	1.03	2.08	1.11	2.50	1.42
Elderly people over 60 years old in the family	0.37	0.48	0.29	0.45	0.34	0.47	0.32	0.44	0.30	0.46
Children over 1 year old in the family	0.62	0.49	0.67	0.47	0.57	0.50	0.72	0.45	0.61	0.49
Trust in organic milk	3.87	1.01	3.50	0.95	3.69	0.89	3.36	1.20	3.71	1.08
The experience of paying attention to organic milk	0.19	0.39	0.26	0.44	0.25	0.43	0.20	0.4	0.18	0.38

*Note.* SD stands for “standard deviation”.

**Table 6:** Logit estimation results of random parameters of the influence of environmental protection information and quality and safety information on purchase intention.

Variables	Control group	Test group	
	No intervention (group *a*)	Environmental protection information intervention (group *b*)	Quality and safety information intervention (group *c*)
Certf	0.7871^*∗∗∗*^ (0.2062)	1.1366^*∗∗∗*^ (0.2153)	1.1959^*∗∗∗*^ (0.2349)
Brand	0.2286^*∗*^ (0.1729)	0.2609^*∗∗*^ (0.1667)	0.5675^*∗∗∗*^ (0.1706)
Origin	0.2331^*∗*^ (0.1738)	0.2850^*∗*^ (0.1675)	0.3217^*∗∗*^ (0.1793)
Price	−0.0870^*∗∗∗*^ (0.0135)	−0.0780^*∗∗∗*^ (0.0125)	−0.0630^*∗∗∗*^ (0.0131)
Gen	0.2836 (0.2006)	0.5652^*∗∗∗*^ (0.1888)	0.6525^*∗∗∗*^ (0.1912)
Age	−0.2308 (0.0925)	−0.0114^*∗*^ (0.0837)	−0.0692^*∗*^ (0.0877)
Edu	0.0259 (0.1390)	0.2314^*∗∗*^ (0.1426)	0.1409^*∗∗*^ (0.1314)
Income	0.5879^*∗*^ (0.0950)	0.4695^*∗∗∗*^ (0.0927)	0.5288 ^*∗∗*^ (0.0910)
n_elder	0.0644 (0.1824)	0.0454^*∗*^ (0.1688)	0.0902 (0.1702)
n_child	0.0418 (0.1716)	0.0046 (0.1610)	0.0774 (0.1645)
Trust	0.1679^*∗∗*^ (0.0880)	0.1373^*∗∗*^ (0.0966)	0.0981^*∗∗*^ (0.0948)
Attention	0.2415 (0.0685)	0.0847 (0.0633)	0.2445^*∗*^ (0.0671)
Log likelihood	−1835	−1790	−1846

*Note.* ^*∗∗∗*^, ^*∗∗*^, and ^*∗*^ indicate significance at levels of 1%, 5%, and 10%, respectively. The numbers in parentheses indicate standard errors.

**Table 7:** Empirical results of the influence of information intervention on purchase intention in the same crowd.

Variable	The second project experiment		The third project experiment	
	Control group	Test group	Control group	Test group
	No intervention (group d)	Environmental protection information intervention (group e)	No intervention (group f)	Quality and safety information intervention (group g)
Certf	1.0932^*∗∗∗*^ (0.1715)	1.0966^*∗∗∗*^ (0.1724)	1.0470^*∗∗∗*^ (0.1709)	1.3020^*∗∗∗*^ (0.1876)
Brand	0.1706 (0.2490)	0.1952^*∗*^ (0.3768)	0.1287 (0.4155)	0.1388^*∗∗*^ (0.3832)
Origin	0.3499^*∗∗*^ (0.4015)	0.3990^*∗∗*^ (0.3506)	0.3072^*∗∗*^ (0.3931)	0.3635^*∗∗*^ (0.3566)
Price	−0.2161^*∗∗∗*^ (0.0548)	−0.2076^*∗∗∗*^ (0.0503)	−0.1794^*∗∗∗*^ (0.0553)	−0.1373^*∗∗∗*^ (0.0505)
Gen	0.0594 (0.2110)	0.0201 (0.2154)	0.0165^*∗*^ (0.2121)	0.0530 (0.2307)
Age	−0.0480 (0.2813)	−0.0216 (0.2765)	−0.0414 (0.2760)	−0.0510 (0.2826)
Edu	0.1666 (0.2852)	0.1957 (0.2883)	0.0743^*∗∗∗*^ (0.2844)	0.0786^*∗∗*^ (0.3079)
Income	0.4521^*∗∗*^ (0.2896)	0.4103^*∗*^ (0.2899)	0.4395^*∗∗*^ (0.2871)	0.4499^*∗*^ (0.3063)
n_elder	0.0386 (0.1373)	0.2537 (0.1328)	0.0297 (0.1339)	0.1400 (0.1285)
n_child	0.1574 (0.1190)	−0.0201 (0.1223)	0.0903 (0.1173)	0.1196 (0.1130)
Trust	0.4430^*∗*^ (0.0885)	0.5477^*∗∗*^ (0.0793)	0.4684^*∗∗∗*^ (0.0854)	0.4994^*∗∗*^ (0.0741)
Attention	0.0118 (0.1716)	0.0246 (0.1610)	0.0074 (0.1645)	0.0064 (0.1636)
Log likelihood	−1763	−1811	−1802	−1732

*Note.* ^*∗∗∗*^, ^*∗∗*^, and ^*∗*^ indicate significance at levels of 1%, 5%, and 10%, respectively. The numbers in parentheses indicate standard errors.

## Data Availability

The dataset used in this paper is available from the corresponding author upon request.
